The article "Roles of Cells from the Arterial Vessel Wall in Atherosclerosis" was published in 2017. Journal: Mediators Inflamm.

# Roles of Cells from the Arterial Vessel Wall in Atherosclerosis

**DOI:** 10.1155/2017/8135934

**Published:** 2017-06-07

**Authors:** Di Wang, Zhiyan Wang, Lili Zhang, Yi Wang

**Affiliations:** Department of Cardiology, Shanghai General Hospital, School of Medicine, Shanghai Jiao Tong University, Shanghai, China

## Abstract

Atherosclerosis has been identified as a chronic inflammatory disease of the arterial vessel wall. Accumulating evidence indicates that different cells from the tunica intima, media, adventitia, and perivascular adipose tissue not only comprise the intact and normal arterial vessel wall but also participate all in the inflammatory response of atherosclerosis via multiple intricate pathways. For instance, endothelial dysfunction has historically been considered to be the initiator of the development of atherosclerosis. The migration and proliferation of smooth muscle cells also play a pivotal role in the progression of atherosclerosis. Additionally, the fibroblasts from the adventitia and adipocytes from perivascular adipose tissue have received considerable attention given their special functions that contribute to atherosclerosis. In addition, numerous types of cytokines produced by different cells from the arterial vessel wall, including endothelium-derived relaxing factors, endothelium-derived contracting factors, tumor necrosis factors, interleukin, adhesion molecules, interferon, and adventitium-derived relaxing factors, have been implicated in atherosclerosis. Herein, we summarize the possible roles of different cells from the entire arterial vessel wall in the pathogenesis of atherosclerosis.

## 1. Introduction

As a major public health issue, atherosclerosis in concert with its related disorders, such as coronary heart diseases, stroke, and peripheral vascular diseases, has been the leading cause of mortality and morbidity worldwide [1, 2]. In the recent years, some of the pioneers have unceasingly devoted themselves to investigate the possible mechanisms implicated in the pathogenesis of atherosclerosis and have made considerable progress, such as the “response to inflammation” theory based on “response to injury” theory [3] and “response to lipoprotein retention” hypothesis [4–6]. In recent years, the concept that atherosclerosis is a chronic inflammatory disease has been extensively accepted [7–10]. In contrast, uncertainty surrounds whether vascular inflammation is transmitted as traditionally thought via “inside to outside” responses emphasizing the indispensable roles of the intima in the progression of atherosclerosis. Alternatively, the new paradigm of an “outside to inside” hypothesis is supported by compelling evidence [11, 12], which predominantly uncovers the functional significance of the tunica intima, adventitia, and perivascular adipose tissue (also called perivascular fat, PVAT).

Additionally, classical doctrine indicates that smooth muscle cells (SMCs) predominantly from the medial have a crucial impact on the development of atherosclerosis based on their migration into the intima and proliferation [13]. Thus, this review will shed light on different cells, including endothelial cells (ECs), SMCs, fibroblasts, and adipocytes from the tunica intima, media, adventitia, and PVAT and their related cytokines, and elucidate how these cells contribute to the pathogenesis of atherosclerosis (Figure 1).

## 2. The Normal Structure of the Arterial Vessel Wall

To the best of our knowledge, some of the large and moderate arteries, such as the aorta and coronary artery, are composed of the tunica intima, the media, and the adventitia encapsulated by perivascular adipose tissue. Longitudinal vascular ECs covering the inner surface of blood vessels are crucial components of the tunica intima and are sequentially exposed to shear stress due to frictional force from the blood flow [14]. The tunica media is saturated with elastic fibers secreted by sparse SMCs in large arteries (also called elastic arteries); nevertheless, the media of moderate arteries (also named muscular arteries) is circumferentially composed of smooth muscle cells side by side together with disseminated elastic fibers and collagen fibers. As the outermost layer of arterial vessel wall, the adventitia consists of fibroblasts, vasa vasorum, nerve endings, and a few resident inflammatory cells in the loose connective tissue [15]. PVAT is located in the outside of the adventitia without any organized barrier to insulate the two, mainly encompassing adipocytes and other infiltrating immune cells, such as macrophages, T cells, fibroblasts, and capillary endothelial cells, as reviewed by Szasz and Webb [16] (Figure 2).

## 3. The Intima in the Development of Atherosclerosis

### 3.1. The Normal Functions of the Intima

As the endocrinal “organ” of the cardiovascular system, ECs mainly consist of the intima with extremely activated metabolism and exceedingly complicated functions. For example, ECs secrete numerous bioactive substances to modulate vascular tone, such as nitric oxide (NO), prostaglandin I_2_ (PGI_2_), and endothelium-derived hyperpolarizing factor (EDHF), which are regarded as endothelium-derived relaxing factors (EDRFs) as well as endothelin 1 (ET-1), thromboxane A_2_ (TXA_2_), angiotensin II (Ang II), and uridine adenosine tetraphosphate (UP_4_A), which belong to endothelium-derived contracting factors (EDCFs). On the one hand, ECs are natural barriers of the blood vessel to maintain the smoothness of the tunica intima to prevent the platelet and leukocyte adhesion and hazardous molecules from invading into arterial vessel wall. On the other hand, the intact endothelium maintains a physiological equilibrium related to the processes of thrombosis via releasing antithrombotic and thrombotic substances and vascular smooth muscle proliferation by constituting the basement membrane of collagen together with the protective layer of SMCs [17]. Interestingly, ECs exert an important effect on the exchange of substances and active transport [18].

### 3.2. Roles of Endothelial Cells in Atherosclerosis

Endothelial dysfunction (ED) is the primary and a crucial step of the development of atherosclerosis. Numerous cardiovascular risk factors, such as obesity and diabetes mellitus, potentially initiate endothelial cell injury, causing ED [19]. Under normal conditions, the endothelium regulates vascular inflammation by secreting NO, whereas a dysfunctional endothelium accelerates reactive oxygen species (ROS) generation and increases vascular inflammation, which is harmful to the vascular system [20]. The damage to the endothelium upsets the balance between vasoconstriction and vasodilation, which is characterized by increased EDCFs, especially ET-1, and reduced EDRFs, mainly NO, and initiates a series of pathophysiologic changes that promote or exacerbate atherosclerosis, including increased vascular permeability to lipoproteins and augmented leukocyte adhesion, platelet aggregation, and generation of cytokines [7]. On the other hand, various inflammatory cytokines, such as tumor necrosis factor *α* (TNF-*α*), interleukin 1 (IL-1), and IL-6, induce the endothelium to express vascular cell adhesion molecule (VCAM), intercellular adhesion molecule (ICAM), monocyte chemoattractant protein 1 (MCP-1), and other chemokines, consequently promoting the adherence and migration of monocytes [21-24]. Once resident in the intima, monocytes acquire characteristics of tissue macrophages. Monocytes augment the expression of scavenger receptor (SR) and then internalize modified lipoproteins. The above processes consequently lead to the formation of foam cells (FCs), which can be regarded as the early atherosclerotic lesion [8]. After the rupture of the atherosclerotic plaque, the physiological balance between antithrombotic and thrombotic substances is disrupted due to the dysfunction of ECs, which leads to increased thrombotic substances (e.g., von Willebrand factor (vWF), TXA_2_) and attenuated antithrombotic substances, such as heparin. These effects facilitate the process of thrombosis, causing devastating consequences [25]. In conclusion, all the above-mentioned factors contribute to atherosclerosis, indicating the indispensable roles of endothelial cells in the progression of atherosclerosis.

## 4. The Media in the Progression of Atherosclerosis

### 4.1. The Normal Roles of the Media

As mentioned previously, the thickness and components of the media between the tunica intima and adventitia depend on the artery type. The elastic fibers characterized by extensibility, mainly forming the media of large arteries, maintain the intact structure and elastic contraction of arteries. However, the media of moderate arteries is circumferentially saturated with smooth muscle cells in a side-by-side arrangement. Owens recommended that the fully differentiated or mature SMCs could express a unique repertoire of contractile proteins (e.g., smooth muscle myosin heavy chain (SM-MHC) or *α*-smooth muscle actin (*α*SMA)), ion channels, and signaling molecules that are required for its contractile function [26]. During vasculogenesis, SMCs also produce high levels of extracellular matrices (ECMs), including collagen, elastin, proteoglycans, cadherins, and integrins that consist of a major portion of the blood vessel mass [27]. In addition, other components of media collagen fibers play a crucial role in connecting and supporting the blood vessel.

### 4.2. Smooth Muscle Cells Contributing to Atherosclerosis

The relationship between SMCs and atherosclerosis has considerably drawn attention since Ross et al. proposed that SMCs have a principal impact on the development of atherosclerosis due to their migration into the intima and proliferation [13]. Interestingly, migrated SMCs are key players in the process of luminal stenosis after the damage of the intima and the internal elastic lamina. Once numerous SMCs migrate to the intima, their excessive proliferation and apoptosis suppression promote extracellular matrix synthesis and lipid deposition, consequently facilitating arterial wall fibrosis and thickening and the luminal stenosis. First, Ruan et al. and Ishikawa et al. demonstrated that human SMCs express numerous lipid uptake receptors, such as low-density lipoprotein receptor (LDLR) and SR, contributing to the formation of myogenic FCs [28, 29]. Second, SMC proliferation can be inhibited by NO, which is a key component of arterial vessel wall remodeling in response to injury, for example, after angioplasty or vein grafting and during atherosclerosis formation [30]. Hou et al. provided new evidence that vasostatin-2 may function as an atherosclerosis-related factor that inhibits cell proliferation and cell adhesion in SMCs, which are associated with the progression of atherosclerosis [31]. In addition, Lang et al. strongly suggested that luteolin suppresses the migration and proliferation of SMCs via downregulating Akt and Src signals [32]. As mentioned above, the migration and proliferation of SMCs are an indispensable pathological process of atherosclerosis. In addition, some of the ECMs released by SMCs strengthen the fibrous cap of the atherosclerotic plaque to protect against plaque rupture and thrombosis [33]. Shankman et al. demonstrated that the contribution of SMCs within atherosclerotic plaques has been extremely neglected and that the transformation of the SMC phenotype mediated by KLF4 is crucial in lesion pathogenesis utilizing a Myh11-CreERT2 ROSA floxed STOP eYFP ApoE^−/−^ mouse model [34]. In addition, a comprehensive review by Doran et al. listed numerous cytokines likely produced by SMCs, such as platelet-derived growth factor (PDGF), transforming growth factor *β* (TGF-*β*), macrophage inhibitory factor (MIF), interferon *γ* (IFN-*γ*), and MCP-1. These cytokines are likely derived from other cells within lesion cells; thus, the concrete functions of these cytokines in the progression of atherosclerosis remain unclear [35].

## 5. The Adventitia Contributing to Atherosclerosis

Recently, the adventitia, which is the outermost layer of arterial vessel wall, has attracted considerable interest given its complex and dynamic roles. Traditionally, the adventitia was regarded as merely an inert physical barrier separating tissues to provide support for blood vessels and a scaffold for the sympathetic nerve system and the vasa vasorum [36]. However, compelling evidence demonstrated that the adventitia plays a critical role in coordinating the progression of atherosclerosis. In 1962, Schwartz and Mitchell demonstrated that the prevalence and degree of the adventitial cellular infiltration closely correlated with the severity of the atherosclerotic plaque [37]. The most common fibroblasts in the adventitia have the capacity of differentiating into myofibroblasts mainly activated by TGF-*β* [38], consequently increasing local expression of inflammatory cytokines and growth factors (GFs) [39, 40]. In addition, Xu et al. demonstrated that the earliest expression of MCP-1 was detected in the adventitial fibroblasts before the formation of intimal lesions after feeding ApoE^−/−^ mice a hyperlipidic diet [41]. On the other hand, adventitial fibroblast nicotinamide adenine dinucleotide phosphate hydrate (NADPH) oxidase-derived ROS is the sensor and messenger for the early development of vascular disease [42]. For example, Liu et al. recommended that NADPH oxidase inhibitors reduced vascular ROS and the medial area via delivering the NADPH oxidase inhibitor gene to the vascular adventitia in C57BL/6 mice [43]. In addition, after the continuous hyperlipidic diet administration, the activated fibroblasts (AFs) derived from ApoE^−/−^ mice displayed augmented NADPH oxidase activity, O2^−^ production, and increased p47phox levels compared with wild-type mice. These effects are associated with increased proliferation and migration of AFs. In addition, p47phox knockout mediated by siRNA decreased the proliferation and migration of AFs in ApoE^−/−^ mice [44]. Additionally, the vasa vasorum promotes blood and oxygen delivery to the arterial vessel wall, thus providing a suitable environment for the development of atherosclerotic plaque and serving as a conduit for trafficking of resident and progenitor cells into the media and intima [45]. Additionally, Hu et al. hypothesized that adventitial transient receptor potential vanilloid type 1 (TRPV1) and sensory C-fibers may play a pivotal role in the adventitia, underscoring the role of the sympathetic nerve system in the development of atherosclerosis [46].

In addition to fibroblasts, some of the lymphocytes accumulate in the adventitia, as supported by the study that demonstrated that the adventitia is a major site of arterial wall inflammation related to lymphocyte infiltration in atherosclerotic arteries [47]. T helper 1 (Th1) cells are proatherogenic cells that secrete proinflammatory cytokines, such as IL-2, TNF-*α*, and IFN-*γ*. In contrast, regulatory T (Treg) cells are atheroprotective cells that release anti-inflammatory cytokines (e.g., IL-4, IL-5, IL-9, IL-10, and IL-13). Th2 cells and Th17 cells are proatherogenic cells and atheroprotective cells. Natural killer T (NKT) cells are proatherogenic cells; however, the mechanism remains unclear. B-1 cells exert antiatherogenic activities via secreting IgM, contributing to the formation of FCs. B-2 cells stimulate Th1 cells and dendritic cells (DCs) to play a proatherogenic role. B-2 cells also secrete IgG, but its proatherogenic role remains to be elucidated. Innate responsive activator (IRA) cells exert proatherogenic activities by releasing granulocyte-macrophage colony-stimulating factor (GM-CSF), which acts on DCs [48] (Figure 3).

## 6. Multiple Roles of Perivascular Adipose Tissue in Atherosclerosis

PVAT is defined as the adipose tissue around the arteries regardless of location [12] located on the outside of adventitia without laminar structures or any organized barrier to separate the two [16]. The old paradigm suggested that PVAT was merely a mechanical and structural support tissue for the blood vessel. More recently, we realized that PVAT not only stores triacylglycerols/triglycerides and free fatty acids (FFAs) participating in energy metabolism but also secretes quantities of adipokines, such as leptin, adiponectin, visfatin, resistin, TNF-*α*, IL-6, IL-8, MCP-1, and plasminogen activator inhibitor 1 (PAI-1), which play indispensable roles in atherosclerosis by mediating SMC migration and proliferation [49], promoting neointimal hyperplasia and formation [50, 51], stimulating inflammation responses and oxidative stress [52], and regulating vascular tone [53] (Figure 4). For instance, Lamers et al. demonstrated that lipid mediators, such as FFAs and adipokines, affect SMC function via inducing augmented proliferation and inflammatory signaling and proposed that the increased fatty acids and adipokines released by PVAT in obesity may disclose the relationships among SMCs dysfunction, vascular inflammation, and atherosclerosis [54]. Additionally, PVAT plays an indispensable role in the inflammatory response to atherosclerosis. The result of proteomic analysis indicated that empirical adipose tissue (EAT) exhibits increased oxidative stress compared with subcutaneous adipose tissue (SAT) in patients with cardiovascular disease, suggesting its possible connection with myocardial stress. Similarly, perivascular visceral fat results in endothelial dysfunction and accelerates atherosclerosis as demonstrated by transplantation of visceral adipose tissue or SAT immediately adjacent to the right common carotid artery in ApoE^−/−^ mice [55]. On the other hand, the idea that elevated levels of leptin may promote neointimal formation was observed in leptin-deficient ob/ob mice with reduced neointimal formation. In addition, Takaoka et al. found that endovascular injury significantly augments proinflammatory adipokines and attenuates adiponectin in a femoral artery wire injury mouse and iliac artery balloon injury rat. In addition, neointimal hyperplasia after vascular injury was reduced via knockout of TNF-*α* with decreased upregulation of proinflammatory adipokines. Regarding the regulation of vascular tone, adventitium-derived relaxing factors (ADRFs), which are currently referred to as PVAT-derived relaxing factors (PVRFs), play a critical role; however, the mechanism is unclear. Ang 1 to 7 may be potential candidates of PVRFs given that Ang 1 to 7 act on the endothelium to cause the release of nitric oxide, which acts as a hyperpolarizing factor through K (Ca) channels to cause relaxation of the blood vessel in rat aorta [56]. Whether others factors, such as adiponectin, leptin, hydrogen sulfate (H_2_S) generated by cystathionine gamma lyase (CSE), and palmitic acid methyl ester (PAME), are PVRF members remains controversial. Taken together, these results all highlight the proatherogrnic role of PVAT in the development of atherosclerosis based on various studies about the antiatherogenic effect of PVAT [57, 58].

## 7. Conclusions

Conclusively, the functional significance of the inflammatory response in atherosclerosis is increasingly conspicuous. However, the complicated pathogenesis of atherosclerosis remains unclear. From our perspective, endothelial dysfunction, SMC migration and proliferation, the transformation of fibroblasts into myofibroblasts, and adipokines produced by PVAT are predominantly implicated in the pathological process of atherosclerosis. We are looking forward to the discovery of positive and effective therapeutic approaches to reduce the incidence and mortality and ameliorate the prognosis of atherosclerosis-related disorders via restoring the normal function of the endothelium or inhibiting the above processes. Of course, in view of some controversial ideas, we should further investigate the possible roles of different cells from the arterial vessel wall in atherosclerosis to provide a solid foundation for therapeutic interventions for atherosclerosis and its associated disorders.

## Figures and Tables

**Figure 1:** Roles of different cells from the arterial vessel wall in atherosclerosis. Different cells, including endothelial cells, smooth muscle cells, fibroblasts, and adipocytes from the tunica intima, media, adventitia, and perivascular adipose tissue and their related cytokines all participate in the inflammatory response of atherosclerosis via multiple intricate pathways. Endothelial dysfunction, smooth muscle cell migration and proliferation, the transformation of fibroblasts into myofibroblasts, and adipokines produced by perivascular adipose tissue are predominantly implicated in the pathological process of atherosclerosis.

**Figure 2:** The normal structure of the arterial vessel wall. The intima, media, adventitia, and perivascular adipose tissue comprise the intact and normal arterial vessel wall. Therefore, cells from the arterial vessel wall mainly consist of endothelial cells, smooth muscle cells, fibroblasts, and adipocytes. Other cells, such as macrophages, dendritic cells, and T cells, also reside in the arterial vessel wall. In addition, the vasa vasorum promotes blood and oxygen delivery to the arterial vessel wall.

**Figure 3:** The effect of T cell or B cell subsets in atherosclerosis. Th0 cells can differentiate into Th1, Th2, Th17, Treg, and NKT cells. Th1 cells are proatherogenic cells that secrete proinflammatory cytokines. NKT cells are also proatherogenic cells, but the mechanism remains unclear. B-2 cells and IRA B cells are both proatherogenic cells, whereas B-1 B cells and Treg cells exert antiatherogenic effects. The effects of Th2 cells and Th17 cells in atherosclerosis remain unclear.

**Figure 4:** Perivascular adipose tissue contributing to atherosclerosis. PVAT plays a pivotal role in atherosclerosis by releasing numerous adipokines, such as leptin, adiponectin, visfatin, resistin, TNF-*α*, IL-6, IL-8, MCP-1, and PAI-1. These adipokines mediate SMC migration and proliferation, also promoting neointimal hyperplasia and formation, stimulating inflammation responses and oxidative stress, and regulating vascular tone, consequently contributing to atherosclerosis.

## Abbreviations

PVAT: Perivascular adipose tissue
SMCs: Smooth muscle cells
ECs: Endothelial cells
NO: Nitric oxide
PGI_2:_: Prostaglandin I_2_
EDHF: Endothelium-derived hyperpolarizing factor
EDRFs: Endothelium-derived relaxing factors
ET-1: Endothelin 1
TXA_2_: Thromboxane A_2_
Ang II: Angiotensin II
UP_4_A: Uridine adenosine tetraphosphate
EDCFs: Endothelium-derived contracting factors
ED: Endothelial dysfunction
ROS: Reactive oxygen species
TNF-*α*: Tumor necrosis factor *α*
IL: Interleukin
VCAM: Vascular cell adhesion molecule
MCP-1: Monocyte chemoattractant protein 1
SR: Scavenger receptor
FCs: Foam cells
vWF: von Willebrand factor
SM-MHC: Smooth muscle myosin heavy chain
*α*SMA: *α*-Smooth muscle-actin
ECMs: Extracellular matrices
LDLR: Low-density lipoprotein receptor
PDGF: Platelet-derived growth factor
TGF-*β*: Transforming growth factor *β*
MIF: Macrophage inhibitory factor
IFN-*γ*: Interferon *γ*
GFs: Growth factors
NADPH: Nicotinamide adenine dinucleotide phosphate hydrate
AFs: Activated fibroblasts
TRPV1: Transient receptor potential vanilloid type 1
Th1: T helper 1
Treg: Regulatory T
NKT: Natural killer T
DCs: Dendritic cells
IRA: Innate responsive activator
GM-CSF: Granulocyte-macrophage colony-stimulating factor
FFAs: Free fatty acids
PAI-1: Plasminogen activator inhibitor 1
EAT: Empirical adipose tissue
SAT: Subcutaneous adipose tissue
ADRFs: Adventitium-derived relaxing factors
PVRFs: PVAT-derived relaxing factors
H_2_S: Hydrogen sulfate
CSE: Cystathionine gamma lyase
PAME: Palmitic acid methyl ester.
